# A potential field segmentation based method for tumor segmentation on multi-parametric MRI of glioma cancer patients

**DOI:** 10.1186/s12880-019-0348-y

**Published:** 2019-06-17

**Authors:** Ranran Sun, Keqiang Wang, Lu Guo, Chengwen Yang, Jie Chen, Yalin Ti, Yu Sa

**Affiliations:** 1 Department of Biomedical Engineering, Tianjin University, 92 Weijin Road, Tianjin, 300072 China; 2 Department of Radiotherapy, Tianjin Medical University General Hospital, Tianjin, 300052 China; 3 Department of Radiation Oncology, Tianjin Cancer Hospital, Tianjin, 300060 China; 4 Global Research Organization, GE Healthcare, Shanghai, 201203 China

**Keywords:** Brain tumor, Functional magnetic resonance imaging, Fusion, Semi-automatic segmentation

## Abstract

**Background:**

Accurate segmentation of brain tumors is vital for the gross tumor volume (GTV) definition in radiotherapy. Functional MR images like apparent diffusion constant (ADC) and fractional anisotropy (FA) images can provide more comprehensive information for sensitive detection of the GTV. We synthesize anatomical and functional MRI for accurate and semi-automatic segmentation of GTVs and improvement of clinical efficiency.

**Methods:**

Four MR image sets including T1-weighted contrast-enhanced (T1C), T2-weighted (T2), apparent diffusion constant (ADC) and fractional anisotropy (FA) images of 5 glioma patients were acquired and registered. A new potential field segmentation (PFS) method was proposed based on the concept of potential field in physics. For T1C, T2 and ADC images, global potential field segmentation (global-PFS) was used on user defined region of interest (ROI) for rough segmentation and then morphologically processed for accurate delineation of the GTV. For FA images, white matter (WM) was removed using local potential field segmentation (local-PFS), and then tumor extent was delineated with region growing and morphological methods. The individual segmentations of multi-parametric images were ensembled into a fused segmentation, considered as final GTV. GTVs were compared with manually delineated ground truth and evaluated with segmentation quality measure (*Q*), Dice’s similarity coefficient (*DSC*) and *Sensitivity* and *Specificity*.

**Results:**

Experimental study with the five patients’ data and new method showed that, the mean values of *Q*, *DSC*, *Sensitivity* and *Specificity* were 0.80 (±0.07), 0.88 (±0.04), 0.92 (±0.01) and 0.88 (±0.05) respectively. The global-PFS used on ROIs of T1C, T2 and ADC images can avoid interferences from skull and other non-tumor areas. Similarity to local-PFS on FA images, it can also reduce the time complexity as compared with the global-PFS on whole image sets.

**Conclusions:**

Efficient and semi-automatic segmentation of the GTV can be achieved with the new method. Combination of anatomical and functional MR images has the potential to provide new methods and ideas for target definition in radiotherapy.

## Background

Gliomas are the most common primary brain tumors in adults which account for 70% of all adult malignant primary brain tumors [1]. The prognosis of therapy is often poor because the tumor preferentially infiltrates into surrounding normal tissue rapidly [2, 3]. Therefore, accurate definition of gross tumor volume (GTV) in radiotherapy is crucial for better prognosis. According to International Commission on Radiation Units & Measurements (ICRU) report No.83, the GTV is the gross demonstrable extent and location of the tumor, may consist of a primary tumor, metastatic regional node(s), or distant metastasis [4]. Magnetic resonance imaging (MRI) has recently become the imaging modality of choice for evaluating tumor progression. In clinical routine, the diagnosis of gliomas relies predominantly on MRI such as T1-weighted contrast-enhanced and T2/fluid attenuated inversion recovery (FLAIR) sequences [5]. Usually, the tumor mass is determined by the enhanced region on contrast-enhanced T1 images, and the peri-tumoral edema is determined by the hyperintensity portion on T2 or FLAIR images, where the possibility of tumor invasion resides [6]. Especially on T2 images, the edema region can appear brighter than those on other MRI sequences [1].

However, the tumor may extend beyond the imageable component in conventional MRI, such as T1C, T2, FLAIR, etc. For instance, high grade gliomas appear to be infiltrating and invading the surrounding tissue along white matter [7]. If these areas can be identified during radiotherapy, it will play a positive role in improving the efficacy of treatment. Therefore, functional MRI techniques which may provide deeper insight about the physiological process of tumors have been investigated to improve the definition of the tumor extent.

It has been proven that apparent diffusion constant (ADC) values, generated from diffusion weighted imaging (DWI), are sensitive to the random water displacement which is related to the cellularity of brain tumors [8]. Also, the necrosis and edema can be identified by higher ADC values compared to the normal tissue [6]. Moreover, diffusion tensor imaging (DTI) is able to model the water diffusion process three-dimensionally, providing better assessment of brain tissue and tumor extent. Based on the fact that tumor leads to a decrease in the directionality of the white matter fiber bundles, fractional anisotropy (FA) values, generated from DTI, could be used to evaluate the tumor infiltration into normal white matter [8]. It has been shown that those functional MRI images are advantageous in providing specific physiological information about tumor progression and could be used to get better definition of the GTV in gliomas than the conventional MRI images [9, 10]. However, images acquired with single parameter alone, either functional or conventional, is not capable of defining the tumor accurately. Integration of both anatomical and functional images seems to be the optimal solution for accurate segmentation of tumor extent. Cai et al. first integrated conventional structural and diffusion tensor MR imaging to distinguish brain tumor tissue types and identified regions of probable abnormality [11]. Kazerooni et al. proposed a multi-parametric brain tumor segmentation approach based on fusion of anatomical and functional images and differentiated various tumorous regions with sensitivity, specificity and dice score all above 80% [6].

Currently, manual segmentation by radiation oncologist is still the routine practice in clinic and used as the ground truth in comparative studies or evaluating algorithms [12, 13]. But it is a tedious and time-consuming task which makes an automated brain tumor segmentation method more desirable [14]. Techniques for automatic segmentation can be roughly divided into conventional methods, classification and clustering methods based on machine learning or deep learning, and deformable model methods. Conventional methods, including threshold-based and region-based methods, are usually hard to achieve satisfactory segmentation results and merely used as a preprocessing step in most situations [15]. Classification and clustering methods are mostly based on machine learning techniques, such as Support Vector Machines [16], Bayesian Classifier [17], Markov Random Fields [18] and Random Forests [19]. Deep learning algorithms also show good application prospects, such as the convolutional neural networks (CNNs) [20]. At the 7th Brain Tumor Segmentation (BraST) challenge organized by Medical Image Computing and Computer Assisted Interventions (MICCAI) in 2018, some new algorithms based on deep learning performed very well on both glioma segmentation and prediction of patient overall survival [21–24]. These methods can model complex relationships or patterns from empirical data and make accurate decisions [15] but usually require a training phase prior to segmenting a set of images [14]. The deformable model methods are usually implemented with other algorithms in most cases due to the requirement of initial contours [15].

There have been publications on study of auto-segmentation of functional images in recent years. For example, Timothy L. Jones et al. applied the K-means method to segment DTI images and the results were considered as biomarkers for tumor classification [25]. However, it is still difficult to accurately segment tumor targets from functional images of poor resolution and lack of sharper edges. Based on the research and analysis of existing algorithms, we proposed a new method analogous to the concept of potential field [26], combining with other algorithms, to segment the GTV on T1C, T2, ADC, FA images separately and obtain final fusion segmentation for glioma cancer patients.

The paper is organized as follows. The detailed segmentations for individual images and ensemble method are described in Section 2. The results and discussion are presented in Section 3 and Section 4. And the conclusions are summarized in Section 5.

## Methods

### Imaging and pre-processing

In this retrospective study, images from 5 patients with gliomas, including 3 high-grade and 2 low-grade were used. T1C images were acquired using fast spin echo sequence with TR/TE = 500/14 ms, image matrix = 512 × 512, field of view = 240x240mm^2^ and slice thickness = 5 mm. T2 images were acquired using fast spin echo sequence with TR/TE = 3900/92 ms, image matrix = 512 × 512, field of view = 240x240mm^2^ and slice thickness = 5 mm. DWI images were acquired using spin-echo echo-planar sequence with TR/TE = 4900/85 ms, image matrix = 256 × 256, field of view = 240x240mm^2^, slice thickness = 6 mm, b-values of 0 and 1000s/mm^2^ in three orthogonal directions. DTI images were acquired using spin-echo echo-planar sequence with TR/TE = 6000/85 ms, image matrix = 256 × 256, field of view = 240x240mm^2^, slice thickness = 6 mm, number of slices = 19, diffusion-sensitizing gradient encoding applied in 25 directions with b value of 1000s/mm^2^, and one image set acquired without diffusion-sensitizing gradients. All images were acquired on a 1.5 T MR scanner (GE Signa Excite) and generated on a GE medical imaging workstation by analyzing the original image sets.

The acquired images of the four parameters differ in resolution and spatial coordinates. Considering the rigid bone of skull confines the brain tissue and leads to little significant non-rigid transformation, three-dimensional (3D) rigid-body registration was used to correct the differences. T2, ADC and FA image sets were adjusted to the same size as the primary image set of T1C with cubic spline interpolation and then mapped to T1C based on mutual information measures. The registration was completed using the Assisted Alignment Method which is an automatic image registration tool of MIM 5.2 (MIM Software Inc., Cleveland, OH) with 6 degrees of freedom and was only intra-patient based on the image grayscale instead of the registration against a template atlas. The Assisted Alignment Method optimized mutual information measures using partial voxel translations and angular rotations which resulted in less than one voxel alignment.

### Segmentation and fusion

Potential field segmentation (PFS), proposed by Cabria et al. to segment brain tumor from FLAIR image, is based on an analogy to the concept of potential field in physics and views the intensity of a pixel in an MRI as a “mass” that creates a potential field. An image is defined as a set of pixels *L* = {*p*_1_, *p*_2_, .. …, *p*_*n*_}, the potential field at pixel *p*_*i*_ (Φ(*p*_*i*_)) is given analogically to Newton’s law of universal gravitation:

1 $$ \Phi \left({p}_i\right)=\sum \limits_{j=1}^n{\Phi}_j\left({p}_i\right)=\sum \limits_{j=1}^n\frac{-{w}_i^2}{{\left\Vert {p}_i-{p}_j\right\Vert}^2} $$

where *p*_*j*_ is all other pixels of the image, *w*_*i*_ is the intensity of pixel *p*_*i*_, ‖*p*_*i*_ − *p*_*j*_‖ is the Euclidean distance between *p*_*i*_ and *p*_*j*_ , and *n* is the total number of image pixels. The potential field calculation is a significant enhancement of the contrast (Fig. 1(b)). And an adaptive potential threshold *t*_ϕ_ is calculated consequently:

2 $$ {t}_{\upphi}={\upphi}_{\mathrm{min}}+\beta \cdot \left({\upphi}_{\mathrm{max}}-{\upphi}_{\mathrm{min}}\right) $$

where ϕ_max_ is the maximum of n potential fields of the image and ϕ_min_ is the minimum. Then every pixel of the image meeting ϕ(*p*_*i*_) ≤ *t*_ϕ_ is associated with the tumor.

**Fig. 1:** The potential fields of one image calculated with two methods. (**a**) original FA image, (**b**) potential field of FA image calculated with Eq. (2), (**c**) potential field of FA image calculated with Eq. (3)

Potential field segmentation (PFS) with a complete image set (global-PFS) is a quadratic-time algorithm with the time complexity expressed as *O*(*n*^2^) since the potential field at *p*_*i*_ is defined as the sum of the individual potentials created by all other pixels. In practice, global-PFS is time-consuming which has disadvantages for clinical use. It can be seen from Eq. (1) that the individual potential field of *p*_*i*_, generated by *p*_*j*_, is significantly reduced with increasing distance between them, so it is reasonable to ignore the potential field generated by pixels farther away. In order to improve the computational efficiency as well as to ensure satisfactory enhancement of image, the local potential field of pixel *p*_*i*_ is calculated instead of the global (Fig. 1 (c)):

3 $$ {\upphi}_{local}\left({p}_i\right)=\sum \limits_{p_j\in {N}_i}{\upphi}_j\left({p}_i\right) $$

where *N*_*i*_ is a *M* × *M* neighborhood of *p*_*i*_. In the calculation of potential field, the efficiency reduces as *M* grows, but the enhancement of image increases. To achieve a balance between these two factors, *M* is set as 5 according to our experimental studies and the verified neighborhood can approximately represent local features. The new segmentation is named as local potential field segmentation (local-PFS). For FA images, local-PFS was used to remove white matter (WM). For T1C, T2 and ADC images, global-PFS was used on partial image including complete tumor.

#### Segmentation for T1C/T2/ADC images

The tumorous regions in T1C, T2 and ADC images appear hyperintense generally, which are similar to those found in FLAIR image (Fig. 2). In T1C, T2, and ADC images, comparing with the contralateral healthy tissue, the abnormal hyperintense region as well as the non-hyperintense regions surrounded by it are both defined as tumors. However, the segmented hyperintense regions include not only brain tumor but also non-cancerous region, such as skull. Therefore, as the first step to extract a hyperintense region, global-PFS was used on a user defined region of interest (ROI) which is a rectangular area that encloses the tumor completely. The segmentation algorithm was coded and implemented with MATLAB, the regional extraction function named as “imcrop” of MATLAB was used. The ROIs were defined slice by slice on the 2D images in a scanned 3D dataset, the same way as radiation oncologists contour ROIs manually. The 3D GTVs were obtained through inter-slices trilinear interpolation after the segmentation. Artifacts produced by this interpolation method were not taken into account. In order to contain unsegmented lesions due to obscure hyperintense and remove non-cancerous regions (Fig. 3 (b), (e) and (h)), a series of sequential morphological image processing was applied on the segmented binary results. Firstly, holes were filled and largest connected area of the results was extracted to remove non-cancerous region. Then morphological opening and closing with a flat disk-shaped structural element of 3 pixels in diameter were successively employed to achieve more smooth boundaries. The results are shown in Fig. 3 (c), (f) and (i).

**Fig. 2:** Multimodal images of a patient with astrocytoma. (**a**) T1-weighted contrast-enhanced image, (**b**) T2-weighted image, (**c**) apparent diffusion coefficient (ADC) image, (**d**) fluid attenuated inversion recovery (FLAIR) image

**Fig. 3:** Segmentation of T1C, T2 and ADC images. (**a**) T1C image, (**b**) segmentation of T1C image by the potential field segmentation, (**c**) final segmentation of T1C, (**d**) T2 image, (**e**) segmentation of T2 image by the potential field segmentation, (**f**) final segmentation of T2, (**g**) ADC image, (**h**) segmentation of ADC image by the potential field segmentation, (**i**) final segmentation of ADC

#### Segmentation of FA images

When the white matter (WM) in brain is displaced or destroyed by tumor infiltrates, the FA value at the original position decreases. Therefore, compared with the contralateral healthy brain tissue, the area with a decreased FA value is identified as tumorous region. With the advantage of segmentation on hyperintense regions, local-PFS was implemented to extract WM in FA images (Fig. 4 (b)). We employed the negation operation to remove WM from FA images and the remaining hypointense region were defined into two parts, a) *R*: the normal area without WM distribution, roughly symmetrical about the midline of brain, and b) the lesion area with tumor or infiltration. The presence of lesions disrupts the symmetry of hypointense region, biasing the center to itself as shown in Fig. 4 (c). Thus, the physical center is calculated to locate tumor and the center (*m*, *n*) is given by:

4 $$ \left(m,n\right)=\arg \min \sum \limits_{\left(i,j\right)\in R}\left|m-i\right|+\left|n-j\right| $$

where (*m*, *n*) and (*i*, *j*) are both pixels belonging to R. With the center m,n as seed (Fig. 4 (d)), region growing was then performed to segment tumorous region.

**Fig. 4:** Segmentation on FA image. (**a**) original FA image, (**b**) segmentation by the potential field segmentation, (**c**) rest of image removing WM, (**d**) locating seeds tumor, (**e**) final segmentation by region growing

The region growing is the simplest and most commonly region-based segmentation method to extract a connected region from an image by selecting initial seed points and utilizing the similarity of seed and adjacent pixels [27]. The initial seed can be chosen manually or automatically [28], and the similarity criteria is determined by a range of pixel intensity values or other features [1]. The procedure terminates when no more pixels agree with the criteria. In this paper, the initial seed is automatically calculated (pixel(*m,n*)), and the similarity criteria is determined by gradient:

5 $$ {G}_g\le \alpha \cdot {G}_s,0.5\le \alpha \le 2 $$

where *G*_*g*_ is the gradient of pixels to be grown, *G*_*s*_ is the gradient of seed point, and *α* is the coefficient controlling the growth range. The sum of horizontal and vertical gradients of a pixel is defined as the actual gradient. Due to the poor resolution and noise of FA images, the gradients of both seed and growth pixels are represented by the average gradient of 3 × 3 neighbors around them to eliminate the obstacles.

Finally, a group of same morphological post-processing steps as performed on T2 and ADC images were added to optimize the grown region and the final result is shown in Fig. 4 (e).

#### Fusion of multiple parametric images

An ensemble approach is proposed to generate a fused segmentation that combines pixel-level information from the segmented results of T1C, T2, ADC and FA images. The segmented images from T1C, T2, ADC and FA images were denoted as *S*_*T*1*C*_, *S*_*T*2_, *S*_*ADC*_ and *S*_*FA*_ separately. The fusion result (denoted as *S*_*multi*_) was produced by the union of individual results:

6 $$ {S}_{multi}={S}_{T1C}\cup {S}_{T2}\cup {S}_{ADC}\cup {S}_{FA} $$

### Evaluation

Calculating the overlap with the ground truth is the most common way to quantitatively evaluate segmentation results [1]. For the segmentation task in 2018 BraTS challenge, manual segmentation labels were used as reference standards [21, 24]. Similarly, referring to the evaluation of most current tumor segmentation algorithms [12, 13, 15], the manual delineation of GTV on the same MR images is considered the ground truth for validation [27]. In this study, the GTV was defined by the radiation oncologists on the image sets slice by slice through visual inspection for each patient. It was performed by one experienced radiation oncologist blinded to the auto-segmented results and was reviewed and validated by another experienced radiation oncologist. On T1C, T2 and ADC images for each patient, GTVs are the whole regions bounded by abnormal hyperintense areas comparing with contralateral normal brain tissues. The GTVs on FA images are the hypointense regions with lower FA values comparing with contralateral normal white matter. Finally, the GTV was generated by the union of each on T1C, T2, ADC and FA.

The segmentation quality measure *Q* was used for quantitative comparisons between manually delineated GTV (denoted as *G*) and semi-automatically segmented GTV (denoted as *S*) of each patient. The parameter *Q* is defined as:

7 $$ Q=\frac{\left|S\cap G\right|}{G}\times \frac{\left|S\cap G\right|}{S} $$

where 0 ≤ *Q* ≤ 1 presents the percentage of pixels in agreement with the ground truth [26]. To evaluate the agreement between the semi-auto segmented and ground truth, Dice’s similarity coefficient (*DSC*) was used [29]:

8 $$ DSC=\frac{2\left(G\cap S\right)}{G+S} $$

DSC Values range from 0 to 1, in which 0 means total disunity of semi-auto and manual segmentation and 1 means equal and total unity in shape of the two. The *Sensitivity* and *Specificity* were calculated as:

9 $$ Sensitivity=\frac{S_{TruePositive}}{S_{TruePositive}+{S}_{FalseNegative}} $$

10 $$ Specificy=\frac{S_{TrueNegative}}{S_{TrueNegative}+{S}_{FalsePositive}} $$

where the *S*_*TruePositive*_ is the intersection of semi-auto and manual segmentation, *S*_*FalseNegative*_ is the area in the manual but not in the semi-auto segmentation, *S*_*TrueNegative*_ is the area not included in either semi-auto or manual segmentation, and *S*_*FalsePositive*_ is the over-segmented area in semi-auto but not included in manual segmentation.

## Results

The new potential field segmentation based algorithm was implemented for segmentation on multi-parametric MRI data of T1C, T2, ADC and FA from five patients. Total number of the images used is 164, which is a reasonable and valid amount of sample images verified with power analysis. The segmented GTVs were compared with manually delineated regions and evaluated with *Q, DSC* and other parameters. Figure 5 illustrates the visual comparison results on multi-parametric images from one of the cases. Figure 6 shows the comparisons of fusion segmentations and GTVs registered on T2 images of five patients. Table 1 lists the corresponding evaluation results of *Q*, *DSC*, *Sensitivit*y and *Specificity*. The *Q* values of all patients are larger than 0.70, ranging from 0.71 to 0.89, comparable or even outperforming the average value (0.612) of FLAIR segmentation obtained with global potential field segmentation (global-PFS) [26]. The *DSC* values are larger than 0.80, ranging from 0.81 to 0.92. The mean *DSC* is 0.88 (±0.04), revealing a high agreement between the semi-auto and the manual segmentation. The mean values of *Sensitivity* and *Specificity* are 0.92 (±0.01) and 0.88 (±0.05), which demonstrate that the GTVs segmented with the new method shows good performance as compared with the manually defined ground truth.

**Fig. 5:** The segmentation results. (**a**) the segmentation of T1C image, (**b**) the segmentation of T2 image, (**c**) the segmentation of ADC image, (**d**) the segmentation of FA image, (**e**) the fusion segmentation presented on T2 image

**Fig. 6:** Comparison between manual and auto segmentation fusion results. The fusion results are showed on axial slices of T2 images of 5 patients (**a** through **e**)

**Table 1:** Evaluation of the semi-auto segmentation results

WHO grade	DSC	Sensitivity	Specificity	Q
II	0.81	0.92	0.86	0.71
II	0.88	0.93	0.81	0.83
III	0.92	0.92	0.88	0.89
IV	0.91	0.93	0.92	0.84
IV	0.86	0.89	0.95	0.73
Mean ± SD	0.88 ± 0.04	0.92 ± 0.01	0.88 ± 0.05	0.80 ± 0.07

*WHO* World Health Organization, *DSC* Dice’s similarity coefficient, *SD* standard deviation

In addition, the improved local-PFS reduced the time complexity from *O*(*n*^2^) to *O*(25 × *n*) and segmentation time from 47 s to less than 1 s for a 512 × 512 FA image, which significantly improves the operational efficiency.

## Discussion

Anatomical and functional MR images could be combined to detect the GTVs for gliomas radiotherapy. Each parameter image has advantages in providing specific information and different image features. However, it is difficult to perform automatic segmentation on multi-parametric images with single method. In this study, a new potential field segmentation based algorithm was developed and applied with other post-processing approaches on multi-parametric MRI data including T1C, T2, ADC and FA to evaluate the feasibility. The results were satisfactory as compared to the ground truth.

Application of the new local-PFS method on FA images reduced the time complexity from *O*(*n*^2^) to *O*(25 × *n*) and ensured the comparable segmentation of image with original calculation of potential field. The combination with other post-processing approaches performed well on segmentation for multi-parametric images. For T1C, T2 and ADC, a series of morphological post-processing steps were added to make up for deficiencies. For FA images, local-PFS was employed to set the initial seed, and then region growing was used to complete the segmentation. In comparison with the current auto segmentation methods, most of which are based on machine learning technique, no training process is needed. The condition of tuning fewer parameters also improves the efficiency and robustness of the segmentation.

Segmentation quality measure with *Q*, *DSC*, *Sensitivity* and *Specificity* demonstrated that satisfactory results could be obtained with the new potential field segmentation based method. The standard deviation of the parameters (< 0.1) showed the robustness of the algorithm. However, the lowest four value of the five parameters appear in the evaluation of low-grade glioma segmentation, probably due to the lower contrast of image compared with high-grade glioma.

In this study, the synthesis of multi-parametric images provides a more accurate and comprehensive reference for GTV definition in radiotherapy. Single parametric image cannot show tumor sufficiently, fusion of multi-parametric images provides more useful information for accurate definition of GTV boundary in radiotherapy which helps in achieving the disease control and better protection of normal tissues at the same time.

It should also be pointed out that for the potential field segmentation algorithm, we only performed experiments on images of glioma patients, and no other body sites or tumor types have been studied. Moreover, the potential field segmentation has not been able to differentiate among neoplasm and edema [30, 31]. Identification of tissues that are likely to progress to neoplasm is also a potential subject for future studies.

## Conclusions

Efficient and automatic segmentation of the GTVs for glioma tumors can be achieved with the new potential field segmentation based multi-parametric MRI segmentation approach which has the potential to accurately segment the tumor regions for target definition in radiotherapy. Further evaluation is needed with more data from glioma patients before clinical application.

## Data Availability

The datasets analyzed during the study are not publicly available due to relevant data protection laws.

## Abbreviations

ADC: Apparent diffusion constant
DTI: Diffusion tensor imaging
DWI: Diffusion-weighted-imaging
FA: Fractional anisotropy
FLAIR: Fluid attenuated inversion recovery
GTV: Gross tumor volume
MRI: Magnetic resonance imaging
PFS: Potential Filed Segmentation
WM: White matter
